# Do Chest Compresses with Mustard or Ginger Affect Warmth Regulation in Healthy Adults? A Randomized Controlled Trial

**DOI:** 10.1155/2022/5034572

**Published:** 2022-07-18

**Authors:** Jan Vagedes, Silja Kuderer, Katrin Vagedes, Henrik Szőke, Matthias Kohl, Stefanie Joos, Florian Beissner, Ursula Wolf

**Affiliations:** ^1^Research Department, ARCIM Institute (Academic Research in Complementary and Integrative Medicine), Im Haberschlai 7, Filderstadt 70794, Germany; ^2^Department of Neonatology, University Hospital Tübingen, Calwerstrasse 7, Tübingen 72076, Germany; ^3^Department of Pediatrics, Filderklinik, Im Haberschlai 7, Filderstadt 70794, Germany; ^4^Department of Integrative Medicine, University of Pécs, Vörösmarty utca 3, Pécs 7623, Hungary; ^5^Institute of Precision Medicine, University Furtwangen, Jakob-Kienzle-Straße 17, Villingen-Schwenningen 78054, Germany; ^6^Institute for General Practice and Interprofessional Care, University Hospital Tübingen, Osianderstraße 5, Tübingen 72076, Germany; ^7^Insula Institute for Integrative Therapy Research, Aronstabweg 2, Hannover 30559, Germany; ^8^Institute of Complementary and Integrative Medicine, University of Bern, Fabrikstrasse 8, Bern 3012, Switzerland

## Abstract

**Background:**

Chest compresses with mustard (MU) or ginger (GI) are a complementary treatment option for respiratory tract infections. However, little is known about their specific thermogenic qualities. This study examines the short-term effects of MU, GI, and chest compresses with warm water only (WA) on measurable and self-perceived body warmth in healthy adults.

**Methods:**

This was a single-center, randomized controlled trial with cross-over design (WA versus MU versus GI). 18 participants (23.7 ± 3.4 years; 66.7% female) received MU, GI, and WA in a random order on three different days with a mean washout period of 13.9 days. Chest compresses were applied to the thoracic back for a maximum of 20 minutes. The primary outcome measure was skin temperature of the posterior trunk (measured by infrared thermography) immediately following removal of the compresses (t1). Secondary outcome measures included skin temperature of the posterior trunk 10 minutes later (t2) and several parameters of self-perceived warmth at t1 and t2 (assessed with the Herdecke Warmth Perception Questionnaire).

**Results:**

Skin temperature of the posterior trunk was significantly higher with MU compared to WA and GI at t1 (*p* < 0.001 for both, primary outcome measure) and t2 (WA versus MU: *p*=0.04, MU versus GI: *p* < 0.01). Self-perceived warmth of the posterior trunk was higher with MU and GI compared to WA at t1 (1.40 ≥ *d* ≥ 1.79) and remained higher with GI at t2 (WA versus GI: *d* = 0.74). The overall warmth perception increased significantly with GI (*d* = 0.69), tended to increase with MU (*d* = 0.54), and did not change with WA (*d* = 0.36) between t0 and t1.

**Conclusions:**

Different effects on warmth regulation were observed when ginger and mustard were applied as chest compresses. Both substances induced self-perceived warming of the posterior trunk, but measurable skin temperature increased only with MU. Further research is needed to examine the duration of these thermogenic effects and how chest compresses with ginger or mustard might be incorporated into practice to influence clinical outcomes in respiratory tract infections.

## 1. Introduction

Respiratory symptoms and diseases are among the most common reasons for consultation in general practice [1]. Acute infections such as the common cold can lead to complications such as sinusitis, otitis media, and pneumonia as well as exacerbations of chronic obstructive pulmonary disease and asthma [2]. Increasingly, patients seek integrative treatment options for respiratory ailments to augment conventional treatments [3].

One integrative health approach for treating respiratory diseases, in addition to others, is based on anthroposophic medicine (AM) [4]. AM treatments include medications administered through oral, intramuscular, intravenous, inhalation, and topical routes of administration, as well as external applications such as chest compresses [5–7]. Warm chest compresses with warm water (hereafter referred to as WA) have been reported to stimulate the warmth balance and are described as strengthening the patients' immune system, activating self-regulatory processes, and reducing susceptibility to new infections [8, 9]. Given their specific pharmacological properties, the addition of ginger (Zingiber officinale) or mustard (Sinapis nigra) to warm chest compresses could offer further benefits in the treatment of respiratory infections [10, 11]. The active phytocompounds of ginger (mainly 6-gingerol and 6-shogaol in addition to further phenolics and flavonoids) [12] have antioxidant, analgesic, and anti-inflammatory effects [12, 13], as well as antipyretic [12, 14], antimicrobial [15], antiviral [16], and immunomodulatory properties [17]. The active ingredient of mustard is allyl isothiocyanate [18, 19], which is purported to have antimicrobial activity [19]. Moreover, when applied externally, both substances were shown to have thermogenic qualities [8, 20, 21] by binding to thermosensitive channels of the transient receptor potential (TRP) family on sensory nerve endings [22–24]. Subsequent release of neuropeptides such as the calcitonin gene-related peptide or substance P triggers myocyte relaxation and vasodilatation [25, 26], which contributes to increased cutaneous blood flow. Interestingly, TRP channels may also be involved in the regulation of immune-inflammatory response [27].

To the best of our knowledge, little research has yet been conducted to analyze the specific thermoregulatory effects of warm chest compresses, specifically when thermogenic substances such as ginger or mustard are added. Stritter et al. recently reported different qualities of warmth and relaxation for chest compresses with added ginger (hereafter referred to as GI) and mustard powder (hereafter referred to as MU) based on qualitative-phenomenological data [8]. Although local skin temperature represents one determinant of skin blood flow, the vasodilator response to local warming corresponds better with heat sensation [28]. Stephens and colleagues reported similar levels of blood flow at sites with similar heat sensation but different actual skin temperature [28]. Hence, the combined application of infrared (IR) thermography and validated questionnaires to assess warmth self-perception is needed to understand the specific thermoregulatory effects of warm chest compresses with thermogenic substances.

This study was designed to investigate the short-term measurable body warmth by IR thermography and self-perceived body warmth generated from WA, MU, and GI. We consider this study to be a fundamental step in identifying the patterns of warmth distribution by which compresses might influence health and well-being, in order to guide more specific clinical application of compresses for respiratory conditions.

## 2. Materials and Methods

### 2.1. Study Design

We conducted a randomized vehicle-controlled clinical study with a three-arm cross-over design comparing the thermogenic effects of WA, MU, and GI on psychophysiological parameters in healthy participants. Data were collected at a German hospital between November 2014 and April 2015. The study protocol was approved by the ethics committee of the University of Tübingen (registry number: 465/2014BO1), registered at ClinicalTrials.gov (NCT02285452), and complied with the CONSORT (Consolidated Standards of Reporting Trials) guidelines [29].

### 2.2. Participants

Participants were recruited through flyers and notices posted at the study hospital. Eligible participants were healthy adults aged 18–40 years who provided written informed consent. Exclusion criteria were infectious diseases (with a core body temperature >38°C), skin injuries on the thorax, hypersensitivity to MU or GI products, heart disease, bronchial asthma, pregnancy, and limited literacy of the German language. Upon meeting the inclusionary criteria, participants indicated their sex, age, weight, and height for the calculation of their body mass index (BMI). After study completion, participants were compensated in the form of a €25 voucher at a local restaurant.

### 2.3. Interventions

Consistent with the cross-over design, each participant received WA, MU, and GI in a random sequence on three different days. The washout period between two consecutive interventions averaged 13.86 ± 13.85 days (mean ± standard deviation, Min = 2, Max = 62 days). The mean total time to complete all three interventions was 27.72 ± 18.16 days (Min = 7, Max = 70 days). Participants were asked to refrain from consuming caffeine and nicotine three hours before the chest compress interventions. Each intervention began with a brief verbal introduction (2 min) and the preparation of the participant for the condition to follow (2 min). Hospital gowns were provided, leaving the feet, forearms, and back uncovered throughout the intervention for observation and data collection.

Participants were then asked to comfortably sit quietly for ten minutes [30] in order to permit their skin temperature to acclimate to the temperature of the room. Once adapted, participants received one of the three chest compresses in a seated position. Compresses were prepared with water heated to 39.9 ± 0.4°C. When preparing GI, 40 grams of powder (Zingiberis rhizome powder, Caesar and Loretz GmbH, Hilden, Germany) was poured into warm water and a cotton cloth (folded into 4–6 layers, approx. 20 × 20 cm) was immersed. For MU, 40 grams of prepared powder (Sinapis nigra seed powder, Caesar & Loretz GmbH, Hilden, Germany) was applied to a paper towel, which was folded into a pack with a cotton cloth (closed in on all sides, approx. 20 × 20 cm) and immersed into warm water. For WA, a cotton cloth was immersed into the warm water, without the addition of any substance. The compresses were carefully wrung out, applied to the thoracic back (between the scapulae or slightly below), and covered with a terry towel. The compresses were held in place by additional, circularly wrapped towels and by leaning against the back of the chair.

The compresses remained on the back for as long as the participants felt comfortable, but no longer than 20 minutes to minimize the potential for any skin irritation or discomfort. The duration of the compress intervention was recorded for each participant and each session. After completing the compress intervention, participants remained seated quietly for ten minutes (resting period). The mean room temperature was 22.6 ± 1.6°C, the humidity was 28.8 ± 2.8%, and the relative air pressure was 997.7 ± 9.5 hPa. To achieve standardization with respect to the circadian rhythm of body temperature, the chest compress interventions were conducted between 1:30 and 7:30 pm.

### 2.4. Outcome Measures

Skin temperature was measured with a high-definition IR camera (FLIR SC660, FLIR Systems, Wilsonville, Oregon/USA, image resolution 640 × 480 pixels, thermal sensitivity <30 mK). Pictures of the upper back (posterior trunk) were taken at a distance of 2 meters between camera and skin. IR images were evaluated with the ThermaCAM™ software to obtain precise measures in degrees centigrade (°C).

The Herdecke Warmth Perception Questionnaire (Herdecker Wärmeempfindungs-Fragebogen, HWPQ) [31, 32] was used to assess self-perceived ratings of warmth for 24 different body parts (Cronbach's *α* = 0.93) and for overall warmth. Warmth was rated on a five-point scale ranging from 0 (cold) to 4 (hot). We combined the warmth perception of adjacent smaller body parts to represent larger regions (corresponding to the locations chosen for our secondary outcome measures). Ratings were averaged to determine warmth perception for the posterior trunk (item upper back), anterior trunk (items chest, abdomen, flanks, and groin), face (items forehead and cheeks), hands (items hands and fingers), and feet (items feet and toes). All 24 HWPQ single items were used to graphically display changes in warmth distribution with WA, MU, and GI over time.

Outcome measures were collected at three times: before the intervention (baseline, t0), immediately after the chest compress intervention (postintervention, t1), and 10 minutes following the completion of the intervention (follow-up, t2). At t1, the IR picture of the posterior trunk was taken 1-2 minutes after removing the compress from the back (without drying the back) and the HWPQ Questionnaire was completed immediately following the IR picture.

Participants were also interviewed about adverse effects, such as skin irritation or burning sensations, at t1 and t2.

#### 2.4.1. Primary and Secondary Outcome Measures

Our primary outcome measure was skin temperature (IR measurement) of the posterior trunk at t1. Secondary outcomes were skin temperature of the posterior trunk (IR) at t2 as well as self-perceived warmth (HWPQ) of the posterior and anterior trunk, face, hands, feet, and overall warmth at t1 and t2. During the planning phase of this study, we gave considerable thought to what might best serve as our primary measure(s) of outcome. We initially intended to designate change in actual skin temperature (prepost-comparison) of the feet, lower legs, hands, and face as primary measure (measured with IR thermography) but changed our focus to the posterior trunk region as the main area of interest. Neither the study design nor sample considerations were altered by this reordering of measurement priorities.

### 2.5. Sample Size

When planning the study, no publications examining the psychophysiological effects of chest compresses containing ginger or mustard powder could be identified and thus no data to estimate the sample size were available. A convenience sample of 18 participants was estimated to be sufficient for our purposes.

### 2.6. Randomization

Based on the three-arm study design (WA versus MU versus GI), six different randomization sequences were possible (a = MU-WA-GI, b = MU-GI-WA, c = WA-GI-MU, d = WA-MU-GI, e = GI-MU-WA, and f = GI-WA-MU). Stratified by sex, the participants were randomly allocated to one of these sequence groups. Sealed, opaque random-assignment envelopes were prepared and selected in the presence of a study nurse at the first appointment. Participants were assigned a study identification number for purposes of confidentially tracking progress over time.

### 2.7. Blinding

Participants were not aware of the allocated chest compress sequence, but study personnel were aware of the sequence. The study nurse applied a room spray containing essential oils to diminish olfactory hints (between t0 and t1). Before each intervention, participants were asked “what kind of substance do you smell?” (response options: MU, GI, eucalyptus, lavender, citrus, and peppermint) in order to verify blinding. Participants were permitted to provide multiple answers. At the follow-up (t2), they were asked “which condition did you receive today?” and they were permitted to choose between MU, GI, and WA.

### 2.8. Statistical Analysis

Statistical analysis was performed with R [33] running in RStudio [34]. To handle missing data, we applied single imputation based on predictive mean matching (R package: mice [35]). A total of 40 imputed datasets were created and averaged to generate single imputation values. Sequence effects for condition order were controlled as described above. The procedure proposed by Wellek and Blettner [36] was applied to assess potential asymmetrical sequence effects (due to interaction of treatment and carry-over effects). We therefore calculated the total (sum) of the initial values (t0) of the primary outcome of all three periods per subject and performed a one-way analysis of variance (ANOVA) with the sequence groups as the factor. In the case of a nonsignificant finding, it would be permitted to pool the sequence groups for the main analysis of intervention effects (WA versus MU versus GI). In accordance with the CONSORT 2010 guidelines, no statistical tests on baseline differences between the randomized groups a–f were conducted [29, 37].

The analysis of our primary outcome measure, skin temperature of the posterior trunk at t1, was performed using a linear mixed-effects model (R package: lme4 [38]), with participants as a random effect and condition (WA, MU, and GI) and time (t0, t1, and t2) as fixed effects. The model was completed by an interaction term between condition and time. In the process of model selection, we compared the model without covariates (model A) with a model considering chest compress duration as covariate (model B). This was accomplished by calculating a likelihood ratio statistic, the Akaike information criterion (AIC), the Bayesian information criterion (BIC), and 95% confidence intervals (CI) for the covariate. Based on these results, the model with better goodness of fit was selected and used in the final analysis. For the latter, post hoc comparisons were conducted (R package: lmerTest [39]) in the case of significant main effects (two-tailed *p* < 0.05) to analyze differences between the conditions (called between-analysis) and changes over time (called within-analysis). Bonferroni correction was applied within these separate analyses to avoid inflating the experiment-wise error rate due to multiple testing. Cohen's effect sizes for correlated samples (*d*) were calculated for the post hoc analyses (R package: effsize [40]).

Secondary outcome measures not derived from the primary analysis are reported descriptively with mean differences between the conditions (between-analysis) and mean changes over time (within-analysis) with 95% CI and Cohen's *d* effect sizes. Potential differences in initial room temperature, water temperature, and humidity were examined using one-way ANOVAs with condition as the factor. To determine differences in chest compress duration between the three conditions, we applied a one-way mixed ANOVA with condition as the fixed effect and subjects as the random effect. Data was cross-checked to assure it conformed to a normal distribution. To check for a potential association between chest compress condition and olfactory perception, the success of blinding was verified using the Cochran-Mantel-Haenszel chi-squared statistics with the total number of olfactory perceptions as confounder.

## 3. Results

### 3.1. Characteristics of Participants

A total of twenty-four individuals responded to the recruitment flyers and were assessed for eligibility. Five decided not to participate (CONSORT flow diagram, Figure 1). Nineteen healthy adult participants were randomized and received the chest compress conditions according to the allocated sequence. However, one participant was discontinued from the study when he was identified as having bronchial asthma and his data were excluded from analysis. Thus, the final analysis included 18 participants. Of these, the majority were women (66.7%, *n* = 12), between 21 and 32 years (23.7 ± 3.4 years) and with a mean BMI of 22.5 ± 3.9 kg/m^2^. Baseline characteristics were similar among the participants (Table 1).

### 3.2. Baseline Room and Compress Conditions

Water temperature, room temperature, and humidity did not differ between the three chest compress conditions (water temperature: *F* (2, 51) = 1.48, *p*=0.24; room temperature: *F* (2, 51) = 2.83, *p*=0.07; humidity: *F* (2, 51) = 3.08, *p*=0.05). However, chest compress duration (MU: 4.3 ± 0.8 min; WA: 19.3 ± 2.8 min, GI: 18.4 ± 3.1 min) differed significantly between conditions (*F* (2, 34) = 208.07, *p* < 0.001). Post hoc analysis revealed significant differences between WA and MU (*p* < 0.001, *d* = 7.24) as well as between MU and GI (*p* < 0.001, *d* = 6.19; nonsignificant difference between WA and GI: *p*=0.30, *d* = 0.28).

### 3.3. Analysis of Possible Carry-Over Effects

The total sums for self-perceived warmth of the posterior trunk did not differ between the six sequence groups at t0 (*F* (5, 12) = 0.60, *p*=0.70). Thus, potential carry-over effects were negligible and the groups were pooled together with regard to the chest compress interventions (WA versus MU versus GI) (*n* = 18).

### 3.4. Model Selection

The likelihood ratio statistic (*X*_diff_^2^ (1) = 0.31, *p*=0.58), the AIC (model A: 404.30, B: 405.99), and BIC (A: 438.26, B: 443.05) pointed to a better data approximation by model A. Hence, we decided to use model A (without covariates) for the primary analysis.

### 3.5. Outcomes and Estimation

Six measurements were excluded from the analysis and replaced with missing imputation because the participants had consumed coffee (*n* = 4) or nicotine (*n* = 1) within three hours prior to the intervention or reported fever with core temperature >38°C (*n* = 1). Hence, a total of 11.11% of the IR and 11.11% of the HWPQ data were missing and were imputed with predictive mean matching. Baseline values of the outcome measures were similar between WA, MU, and GI (Tables 2 and 3).

#### 3.5.1. Changes in Measured Skin Temperature (Posterior Trunk)

The primary analysis yielded significant main effects of condition (*F* (2, 136) = 12.72, *p* < 0.001) and time (*F* (2, 136) = 7.84, *p* < 0.001) as well as a significant interaction effect between condition and time (*F* (2, 136) = 7.12, *p* < 0.001). Post hoc analyses revealed that the primary outcome measure, skin temperature of the posterior trunk at t1, was significantly higher with MU compared to WA and GI (Table 2). At t2, skin temperature was still higher after MU compared to WA and GI (Table 2). Skin temperature increased only with MU over time, while it initially decreased with GI and did not change with WA (Table 2 and Figures 2 and 3).

#### 3.5.2. Changes in Self-Perceived Warmth (HWPQ)

*(1) Posterior Trunk*. At t1, self-perceived warmth of the posterior trunk was significantly higher with MU and GI compared to WA and remained higher with GI at t2. No differences were found between GI and MU (Table 3), as self-perceived warmth increased significantly in both conditions over time (Table 4). The comparison of measured (IR) and self-perceived warmth of the posterior trunk indicated consistent courses for MU (increase of warmth) and WA (unchanging warmth) but an inconsistent course for GI (decrease in skin temperature but increase in self-perceived warmth of the posterior trunk) (Figure 2).

*(2) Anterior Trunk*. At t1, self-perceived warmth of the anterior trunk was significantly higher with GI compared to WA. No significant differences were found between WA and MU or between MU and GI (Table 3), nor were there any significant changes over time (Table 4).

*(3) Face, Hands, and Feet*. Self-perceived warmth of the face, hands, and feet did not differ between WA, MU, and GI (Table 3). The descriptive within-analysis yielded a significant decrease in self-perceived warmth of the feet with WA and MU over time (Table 4).

*(4) Overall Warmth*. At t1, highest values for overall warmth were observed with MU and GI (Table 3) with a statistically significant increase from t0 to t1 only with GI (Table 4). The warmth distribution of HWPQ single items indicated a higher perceived warming with GI and MU than with WA (Figure 4).

### 3.6. Success of Blinding

At t0, the correct substance was identified in four (MU: *n* = 1, GI: *n* = 3) of the 54 chest compresses administered (each participant received all three conditions). The most frequent olfactory perceptions were citrus (*n* = 42), eucalyptus (*n* = 12), and lavender (*n* = 6). We found no significant association between GI and ginger olfactory perceptions (Mantel-Haenszel *X*^2^ (1) = 1.07, *p*=0.30) or between MU and mustard olfactory perceptions (Mantel-Haenszel *X*^*2*^(1) = 0.04, *p*=0.84). Thus, at t0, success of blinding can be assumed. At t1, the condition was correctly identified in 44 of 54 possible cases (MU: *n* = 18, GI: *n* = 15, WA: *n* = 11), indicating that the participants were no longer blinded from this point on.

### 3.7. Adverse Effects

Two adverse effects, pruritus (WA: *n* = 1) and headache (GI: *n* = 1), were recorded, but no medical treatment was required.

## 4. Discussion

Our findings demonstrate that chest compresses with ginger and mustard powder have different effects on skin temperature and warmth perception than those with warm water only. MU induced a warming effect in both IR thermography and warmth perception of the posterior trunk, whereas GI had a mixed effect with measurable skin temperature cooling (posterior trunk) but a stronger self-perceived warming (posterior and anterior trunk). The influence of WA on skin temperature and warmth perception was negligibly low. After all chest compresses, the self-perceived warmth spread mainly throughout the upper body, while the extremities tended to be perceived as cooler.

WA did not demonstrate significant effects on warmth regulation in healthy adults; however, the addition of ginger or mustard powder was an activating component for the thermogenic efficacy of chest compresses. This might be associated with the activation of TRP channels on sensory nerve endings by the active ingredients of ginger and mustard [22–24]. Moreover, the distinct TRP activation pattern may explain the different effects of both substances on skin temperature and warmth perception. Shogaols and gingerols, the active ingredients of ginger, primarily activate the TRP vanilloid receptor 1 (TRPV1) [22, 24], which is classified as a heat receptor [41]. Allyl isothiocyanate, the active ingredient of mustard, also activates TRP ankyrin 1 (TRPA1) [23], which is classified as a cold receptor [41]. Since TRP channels are key players in early thermosensation transduction [41], the exclusive activation of heat receptors by ginger could explain the higher and longer-lasting effect of ginger on warmth perception [20, 21]. In our study, the self-perceived warmth encompassed the anterior trunk, face, and hands, and the overall warmth increased with GI. With MU, the self-perceived warmth was experienced mainly in the trunk, but the limbs were perceived as colder. Our findings are consistent with those of Stritter et al., in which participants reported mainly a warming effect that spread throughout the body when ginger powder was added to chest compresses and more relaxing effects when mustard powder was used [8].

Interestingly, in our study, the self-perceived warmth generation of GI did not necessarily coincide with the measured skin temperature. The autonomic response to an exogenous heat application includes cutaneous vasodilatation to allow radiant and convective heat loss [42]. Therefore, an increase in the skin temperature of the posterior trunk would have been expected after all three chest compress interventions (not only after MU). Beyond that, the active ingredients of ginger and mustard also have vasodilatory effects [25, 26]. It could be hypothesized that MU has a stronger effect on the skin surface, which can be mapped by IR thermography (penetration depth of IR thermography∼3–5 mm), whereas GI extends to deeper tissue layers and affects the self-perception of warmth more (which would not be measured by IR thermography). However, the participant-determined chest compress duration was significantly shorter for MU than for GI and WA. It therefore remains to be clarified whether a specific substance effect or the duration of the compresses or both lead to the differing effects of the compresses on skin temperature. Since the prolonged topical application of mustard may lead to severe adverse skin reaction [23, 24, 43, 44], immediate discontinuation of the chest compress intervention was imperative when participants felt discomfort. In our study, we had two incidents of adverse effects, pruritus (after WA, presumably due to the heat of the water or due to the materials used) and headache (after GI, presumably due to vasoactive processes). Neither event required medical treatment or discontinuation of study participation. No statistically significant differences in the room conditions were found across the three different chest compress interventions and, therefore, room conditions as potential influencing factors can be regarded as negligible.

In anthroposophic medicine, MU and GI are used in the treatment of respiratory infections [8]. GI is traditionally used to treat chronic inflammation of the airways with little secretion [8, 15] as well as for strong, irritable cough (secretolytic effect) [11]. By contrast, MU is traditionally applied for acute inflammation of the airways with obstruction, heavy secretion, and fever (mucolytic effect) [8, 11]. Interestingly, both heat itself and the substance ginger have been described to upregulate the synthesis of heat shock proteins [14, 45]. These molecular chaperones are involved in cellular recovery [14] and in the induction of cytokine secretion, cross-presentation, and T-cell stimulation [46]. The results of the present study suggest different warmth-generating properties of ginger and mustard powder when administered via chest compresses. This observation could serve as a basis and justification for an indication specific application for respiratory disorders.

A range of herbal medicines are progressively used to treat respiratory infections and inflammatory diseases [47, 48], yet whether other plants would evoke more beneficial effects than ginger or mustard when applied as chest compresses still requires investigation. Interestingly, most plants with anti-inflammatory and antioxidant properties produce flavonoid compounds with phenolic structures [49, 50]. Promising results are reported for catechins, the polyphenolic flavonoids of green tea [49], which provide antiviral, antibacterial, anti-inflammatory, and antioxidant activities [51]. Scientific evidence suggests a pathogenic role of free radical damage in respiratory tract infections, which is why substances with antioxidant activity can help to reduce both oxidative stress and inflammation [51]. Further promising plants include *Ophiorrhiza rugosa* [48] and plants of the *Gynura* species [52]. However, the effect of these plants on respiratory tract infections after topical application has not yet been examined. One of the major catechins of green tea, epigallocatechin-3-gallate (EGCG), was shown to be poorly absorbed systemically after topical application [53].

This study was carried out in healthy adults for feasibility reasons. Physical response and self-perceived warmth may differ in patients with acute illness or chronic disease. Therefore, effects of chest compresses on physiological parameters of patients with respiratory diseases and on the course of disease should also be evaluated to understand the potential more fully for chest compress use in respiratory infections and conditions.

Regarding limitations of our study, we enrolled a small sample size of relatively young adult participants. We did not include thermographic measurements of additional body regions (feet, hands, face) or measurement of the body core temperature, and these measurements could contribute to the evaluation of specific effects of chest compresses on the warmth balance. The HWPQ questionnaire is currently the only available instrument for the assessment of warmth perceptions, but the validity of the instrument has not yet been established, although the instrument has been utilized in several published studies [20, 21, 54, 55]. As in our previous studies [20, 21], we were not able to blind the sensory experience of the chest compress conditions when applied directly to the skin. The unblinding of the majority of participants at t2 might have biased the data on self-perceived warmth. In addition, it would be desirable to investigate the effects of regular chest compress applications.

## 5. Conclusion

Chest compresses with ginger and mustard powder have specific warmth inducing qualities when applied to the skin. Mustard appears to increase skin temperature and self-perceived warmth perception, whereas ginger appears to generate higher and longer-lasting self-perceived warming at the treated area. The duration of the warming effect of both substances beyond WA remains unknown. Further research is desirable to clarify whether the different thermogenic effects of ginger and mustard alter the outcome of clinical parameters in patients with respiratory infections and conditions.

## Figures and Tables

**Figure 1:** CONSORT flow diagram. WA, chest compress with warm water only; GI, chest compress with ginger; MU, chest compress with mustard. ^*∗*^Same participant.

**Figure 2:** (a) Infrared thermography. (b) Self-perceived warmth (HWPQ).

**Figure 3:** Skin temperature of the posterior trunk of a female participant in dependence of the compress received. Note: The shown skin temperature (measured with infrared thermography) changes are approximate. The mean changes of the entire participant are collective and are therefore representative. The dark L-shaped structures mark the position of the compresses at the back.

**Figure 4:** Warmth perception assessed with the Herdecke Warmth Perception Questionnaire (HWPQ).

**Table 1:** Baseline (t0) characteristics.

Group (number), chest compress sequence	*a* (*n* = 3), MU-WA-GI	*b* (*n* = 3), MU-GI-WA	*c* (*n* = 3), WA-GI-MU	*d* (*n* = 3), WA-MU-GI	*e* (*n* = 3), GI-MU-WA	*f* (*n* = 3), GI-WA-MU
Demographics						
Age (years)	23.00 ± 1.00	22.67 ± 0.58	23.33 ± 2.52	27.00 ± 5.00	21.67 ± 0.58	24.67 ± 6.35
BMI (kg/m^2^)	23.24 ± 0.82	20.63 ± 0.94	19.76 ± 0.99	25.22 ± 4.97	26.31 ± 6.65	20.00 ± 0.74
Female sex, *n* (%)	2 (66.67)	2 (66.67)	2 (66.67)	2 (66.67)	2 (66.67)	2 (66.67)
Skin temperature (IR) (°C)						
Posterior trunk	34.97 ± 0.50	35.44 ± 0.42	35.59 ± 0.26	35.42 ± 0.62	34.33 ± 1.58	35.69 ± 0.22
Self-perceived warmth (HWPQ) (0 = cold, 4 = hot)						
Posterior trunk	2.33 ± 0.71	2.67 ± 0.71	2.00 ± 0.71	2.33 ± 0.71	2.67 ± 1.12	2.33 ± 0.71
Anterior trunk	2.17 ± 0.45	2.81 ± 0.27	2.22 ± 0.49	2.36 ± 0.31	2.86 ± 0.72	2.36 ± 0.42
Face	2.78 ± 0.36	2.83 ± 0.50	2.22 ± 0.44	2.39 ± 0.55	2.61 ± 1.05	2.67 ± 0.35
Hands	3.11 ± 0.33	2.78 ± 0.36	2.44 ± 0.46	2.56 ± 0.58	3.11 ± 0.33	2.11 ± 0.78
Feet	2.50 ± 0.97	2.00 ± 0.87	2.06 ± 0.63	2.28 ± 0.62	2.00 ± 1.27	1.56 ± 0.73
Overall warmth	2.78 ± 0.44	2.67 ± 0.50	2.33 ± 0.50	2.33 ± 0.71	3.00 ± 0.50	2.44 ± 0.53

Data are means ± SD if not otherwise indicated. WA, chest compress with warm water only; GI, chest compress with ginger; MU, chest compress with mustard; IR, infrared thermography; HWPQ, Herdecke Warmth Perception Questionnaire.

**Table 2:** Post hoc analyses for the primary analysis of skin temperature (infrared thermography) of the posterior trunk.

Mean ± SD				Post hoc analyses for between-differences		

Time	WA	MU	GI	ΔWA vs. MU	ΔWA vs. GI	ΔMU vs. GI

t0	35.26 ± 1.09	35.13 ± 0.85	35.32 ± 0.62	*t* (136) = 0.84, *P*=1.00, *d* = 0.13	*t* (136) = −0.46, *P*=1.00, *d* = 0.08	*t* (136) = −1.30, *P*=1.00, *d* = 0.26

t1	34.99 ± 0.66	35.66 ± 0.55	34.84 ± 0.48	*t* (136) = 4.59, **P** < 0.001, *d* = 1.10	*t* (136) = 1.02, *P*=1.00, *d* = 0.26	*t* (136) = 5.62, **P** < 0.001, *d* = 1.58

t2	35.37 ± 0.65	35.82 ± 0.49	35.26 ± 0.38	*t* (136) = 3.04, **P**=0.042, *d* = 0.77	*t* (136) = 0.79, *P*=1.00, *d* = 0.22	*t* (136) = 3.83, **P** < 0.01, *d* = 1.28

Post hoc analyses for within-changes						

Δt0 vs. t1	*t* (136) = −1.86, *P*=0.98, *d* = 0.30	*t* (136) = 3.58, **P** < 0.01, *d* = 0.73	*t* (136) = −3.34, **P**=0.011, *d* = 0.88			

Δt0 vs. t2	*t* (136) = 0.78, *P*=1.00, *d* = 0.13	*t* (136) = 4.66, **P** < 0.001, *d* = 0.98	*t* (136) = −0.47, *P*=1.00, *d* = 0.14			

WA, chest compress with warm water only; GI, chest compress with ginger; MU, chest compress with mustard; t0, baseline; t1, postintervention; t2, follow-up; *d*, Cohen's *d* effect size. Bold indicates *p* values <0.05.

**Table 3:** Mean values (±standard deviations) and descriptive between-group differences for self-perceived warmth (Herdecke Warmth Perception Questionnaire, HWPQ).

Outcome	Time	Mean ± SD			Mean difference (95% CI); ES		
		WA	MU	GI	ΔWA vs. MU	ΔWA vs. GI	ΔMU vs. GI
Posterior trunk	t0	2.50 ± 0.71	2.39 ± 0.70	2.28 ± 0.96	0.11 (−0.36; 0.59); 0.16	0.22 (−0.35; 0.79); 0.26	0.11 (−0.46; 0.68); 0.13
	t1	2.11 ± 0.96	3.33 ± 0.77	3.56 ± 0.62	**−1.22** (−1.81;−0.63); 1.40	**−1.44** (−2.00;−0.89); 1.79	−0.22 (−0.69; 0.25); 0.32
	t2	2.33 ± 0.84	2.72 ± 0.67	2.94 ± 0.80	−0.39 (−0.90; 0.13); 0.51	**−0.61** (−1.17;−0.05); 0.74	−0.22 (−0.72; 0.28); 0.30

Anterior trunk	t0	2.56 ± 0.52	2.42 ± 0.47	2.42 ± 0.59	0.14 (−0.20; 0.47); 0.28	0.14 (−0.24; 0.51); 0.25	0.00 (−0.36; 0.36); 0.00
	t1	2.33 ± 0.45	2.61 ± 0.49	2.69 ± 0.50	−0.28 (−0.60; 0.04); 0.59	**−0.36** (−0.69;−0.04); 0.75	−0.08 (−0.42; 0.25); 0.17
	t2	2.43 ± 0.37	2.67 ± 0.40	2.72 ± 0.54	−0.24 (−0.50; 0.03); 0.61	−0.29 (−0.61; 0.02); 0.63	−0.06 (−0.38; 0.27); 0.12

Face	t0	2.58 ± 0.69	2.67 ± 0.59	2.50 ± 0.54	−0.08 (−0.52; 0.35); 0.13	0.08 (−0.34; 0.51); 0.13	0.17 (−0.22; 0.55); 0.29
	t1	2.64 ± 0.76	2.58 ± 0.62	2.69 ± 0.57	0.06 (−0.42; 0.53); 0.08	−0.06 (−0.51; 0.40); 0.08	−0.11 (−0.52; 0.29); 0.19
	t2	2.47 ± 0.79	2.81 ± 0.62	2.86 ± 0.41	−0.33 (−0.82; 0.15); 0.47	−0.39 (−0.82; 0.05); 0.61	−0.06 (−0.42; 0.30); 0.11

Hands	t0	2.75 ± 0.43	2.61 ± 0.61	2.69 ± 0.75	0.14 (−0.22; 0.50); 0.26	0.06 (−0.36; 0.47); 0.09	−0.08 (−0.55; 0.38); 0.12
	t1	2.50 ± 0.62	2.28 ± 0.75	2.69 ± 0.82	0.22 (−0.24; 0.69); 0.32	−0.19 (−0.69; 0.30); 0.27	−0.42 (−0.95; 0.12); 0.53
	t2	2.36 ± 0.78	2.28 ± 0.69	2.75 ± 0.73	0.08 (−0.42; 0.58); 0.11	−0.39 (−0.90; 0.12); 0.51	−0.47 (−0.95; 0.01); 0.66

Feet	t0	2.31 ± 0.82	1.83 ± 0.79	2.06 ± 1.01	0.47 (−0.07; 1.02); 0.59	0.25 (−0.38; 0.88); 0.27	−0.22 (−0.84; 0.39); 0.25
	t1	1.72 ± 0.97	1.67 ± 0.80	1.83 ± 0.94	0.06 (−0.55; 0.66); 0.06	−0.11 (−0.76; 0.54); 0.12	−0.17 (−0.76; 0.43); 0.19
	t2	1.42 ± 0.65	1.22 ± 0.73	1.56 ± 0.94	0.19 (−0.27; 0.66); 0.28	−0.14 (−0.69; 0.41); 0.17	−0.33 (−0.90; 0.24); 0.40

Overall warmth	t0	2.67 ± 0.69	2.67 ± 0.49	2.44 ± 0.51	0.00 (−0.40; 0.40); 0.00	0.22 (−0.19; 0.63); 0.37	0.22 (−0.12; 0.56); 0.45
	t1	2.39 ± 0.85	2.89 ± 0.32	2.83 ± 0.62	**−0.50** (−0.94;−0.06); 0.78	−0.44 (−0.95; 0.06); 0.60	0.06 (−0.28; 0.39); 0.11
	t2	2.33 ± 0.91	2.72 ± 0.46	2.56 ± 0.62	−0.39 (−0.88; 0.10); 0.54	−0.22 (−0.75; 0.31); 0.29	0.17 (−0.20; 0.54); 0.31

WA, chest compress with warm water only, GI: chest compress with ginger; MU, chest compress with mustard; t0, baseline; t1, postintervention; t2, follow-up; CI, confidence intervals; ES, Cohen's *d*. HWPQ scores range from 0 = cold to 4 = hot. Bold indicates CI that do not contain zero.

**Table 4:** Descriptive within-group changes from baseline (t0) to postintervention (t1) and from baseline to follow-up (t2) for self-perceived warmth (Herdecke Warmth Perception Questionnaire, HWPQ).

Outcome		Δt1 − t0			Δt2 − t0		
	CD	Diff	CI	ES	Diff	CI	ES
Posterior trunk	WA	−0.39	(−0.96; 0.18)	0.46	−0.17	(−0.52; 0.18)	0.21
	MU	**0.94**	(0.45; 1.44)	1.29	0.33	(−0.08; 0.75)	0.49
	GI	**1.28**	(0.67; 1.89)	1.59	0.67	(−0.02; 1.35)	0.75

Anterior trunk	WA	−0.22	(−0.57; 0.12)	0.46	−0.12	(−0.41; 0.16)	0.28
	MU	0.19	(−0.05; 0.44)	0.40	0.25	(−0.04; 0.54)	0.57
	GI	0.28	(−0.03; 0.59)	0.51	0.31	(−0.01; 0.62)	0.54

Face	WA	0.06	(−0.32; 0.44)	0.08	−0.11	(−0.48; 0.26)	0.15
	MU	−0.08	(−0.43; 0.26)	0.14	0.14	(−0.13; 0.41)	0.23
	GI	0.19	(−0.09; 0.48)	0.35	**0.36**	(0.04; 0.68)	0.75

Hands	WA	−0.25	(−0.55; 0.05)	0.47	−0.39	(−0.83; 0.05)	0.62
	MU	−0.33	(−0.75; 0.08)	0.49	−0.33	(−0.70; 0.03)	0.51
	GI	0.00	(−0.38; 0.38)	0.00	0.06	(−0.21; 0.32)	0.07

Feet	WA	**−0.58**	(−1.07;−0.10)	0.65	**−0.89**	(−1.37; −0.41)	1.20
	MU	−0.17	(−0.53; 0.20)	0.21	**−0.61**	(−1.03;−0.20)	0.80
	GI	−0.22	(−0.71; 0.27)	0.23	−0.50	(−1.18; 0.18)	0.51

Overall warmth	WA	−0.28	(−0.81; 0.26)	0.36	−0.33	(−0.92; 0.26)	0.41
	MU	0.22	(−0.05; 0.49)	0.54	0.06	(−0.21; 0.32)	0.12
	GI	**0.39**	(0.09; 0.69)	0.69	0.11	(−0.23; 0.45)	0.20

CD, condition; WA, chest compress with warm water only; GI, chest compress with ginger; MU, chest compress with mustard; Diff, mean difference; CI, confidence intervals; ES, Cohen's *d* effect size. HWPQ scores range from 0 = cold to 4 = hot. Bold indicates CI that do not contain zero.

## Data Availability

The datasets and materials used during this study are available from the corresponding author upon reasonable request after August 2023.
